The article "Ascertaining yield and grain protein content stability in wheat genotypes having the Gpc-B1 gene using univariate, multivariate, and correlation analysis" was published in 2022. Journal: Front Genet.

# Ascertaining yield and grain protein content stability in wheat genotypes having the *Gpc-B1* gene using univariate, multivariate, and correlation analysis

**DOI:** 10.3389/fgene.2022.1001904

**Published:** 2022-09-07

**Authors:** Mohammad Jafar Tanin, Achla Sharma, Dinesh Kumar Saini, Satinder Singh, Lenika Kashyap, Puja Srivastava, G. S. Mavi, Satinder Kaur, Vijay Kumar, Vineet Kumar, Gomti Grover, Parveen Chhuneja, V. S. Sohu

**Affiliations:** ^1^ Department of Plant Breeding and Genetics, Punjab Agricultural University, Ludhiana, India; ^2^ School of Agricultural Biotechnology, Punjab Agricultural University, Ludhiana, India

**Keywords:** grain protein content, stability analysis, G × E interaction, univariate analysis, multivariate analysis, wheat

## Abstract

The high performance and stability of wheat genotypes for yield, grain protein content (GPC), and other desirable traits are critical for varietal development and food and nutritional security. Likewise, the genotype by environment (G × E) interaction (GEI) should be thoroughly investigated and favorably utilized whenever genotype selection decisions are made. The present study was planned with the following two major objectives: 1) determination of GEI for some advanced wheat genotypes across four locations (Ludhiana, Ballowal, Patiala, and Bathinda) of Punjab, India; and 2) selection of the best genotypes with high GPC and yield in various environments. Different univariate [Eberhart and Ruessll’s models; Perkins and Jinks’ models; Wrike’s Ecovalence; and Francis and Kannenberg’s models], multivariate (AMMI and GGE biplot), and correlation analyses were used to interpret the data from the multi-environmental trial (MET). Consequently, both the univariate and multivariate analyses provided almost similar results regarding the top-performing and stable genotypes. The analysis of variance revealed that variation due to environment, genotype, and GEI was highly significant at the 0.01 and 0.001 levels of significance for all studied traits. The days to flowering, plant height, spikelets per spike, grain per spike, days to maturity, and 1000-grain weight were specifically affected by the environment, whereas yield was mainly affected by the environment and GEI. Genotypes, on the other hand, had a greater impact on the GPC than environmental conditions. As a result, a multi-environmental investigation was necessary to identify the GEI for wheat genotype selection because the GEI was very significant for all of the evaluated traits. Yield, 1000-grain weight, spikelet per spike, and days to maturity were observed to have positive correlations, implying the feasibility of their simultaneous selection for yield enhancement. However, GPC was observed to have a negative correlation with yield. Patiala was found to be the most discriminating environment for both yield and GPC and also the most effective representative environment for GPC, whereas Ludhiana was found to be the most effective representative environment for yield. Eventually, two NILs (BWL7508, and BWL7511) were selected as the top across all environments for both yield and GPC.

The article "Ascertaining yield and grain protein content stability in wheat genotypes having the Gpc-B1 gene using univariate, multivariate, and correlation analysis" was published in 2022. Journal: Front Genet.

## Introduction

Bread wheat (*Triticum aestivum L* *.*) is considered to be the most valuable source of calories and protein across the world (Pal et al., 2022). It is widely grown in different parts of the world, including India, where it is an important staple crop, particularly in the northern region (mainly Punjab State). In many studies, grain protein content (GPC) has been observed to be the most important factor influencing end-use quality and thus has a significant impact on the economic importance of wheat (Saini et al., 2020). As a direct consequence, GPC improvement in wheat has become a top priority in wheat breeding research projects, particularly for those looking at improvement in nutritional quality (Shewry, 2009; Gudi et al., 2022), especially for the people who cannot afford supplements to fulfill their daily recommended intake of protein. Since a negative association is generally observed between GPC and grain yield, developing an elite wheat cultivar having higher yield potential and GPC is considered a major challenge, taking the current growing rate of food requirements into consideration. Breeders can target desirable stable genotypes having high yield potential and GPC based on the results of selection in different environments and more advanced approaches such as genomic selection (Sandhu et al., 2021a, 2021b; Gill et al., 2021, 2022; Saini et al., 2022). Biotic as well as abiotic stresses usually play a considerable role in grain yield and GPC fluctuations, which are closely associated with the immediate response of cultivars to environmental changes (Verma et al., 2015). This type of inconsistency or alteration is known as genotype by environment interaction (GEI), and it has been observed in several crops, including wheat (Ahmed et al., 2011; Mengesha et al., 2019; Ahakpaz et al., 2021).

Wheat breeders have always faced difficulty integrating both high grain yield and high GPC into individual wheat genotypes, mainly because of the following factors: 1) grain yield and GPC are highly influenced by the environment; 2) GPC and grain yield typically have a negative correlation with each other; and 3) both yield and GPC have low to moderate level of heritability and are controlled by a large number of genes (Khazratkulova et al., 2015). Further, the wide range of environmental dependent variables that are available in wheat growing regions brings up the idea that there might be a strong directional interaction present between genotype and environment. This interaction, therefore, occurs whenever the yield potential of individual plant is significantly influenced by the environment in which they are evaluated (Malosetti et al., 2013). To study GEI, two major steps are always considered to be performed: 1) phenotypic characterization of the germplasm in a multi-location trial, which subsequently demonstrates the possible existence of environmental diversity available in growing regions; and 2) analysis of the observed data to explain the structure of the current interaction between genotype and environment and consequently to display the possible environmental-related parameters that help predict the behavior of genotypes in untested environments (Hilmarsson and Roi, 2021). As a result, rather than selecting according to the average performance of cultivars conferring a wider level of adaptation, it is preferred to arrange environments with identical G x E performances into mega-environments to select individual plants conferring local adaptations to different environmental circumstances (Gauch and Zobel, 1997; Gauch, 2013). Moreover, designing a multi-environmental trial to verify the stability and performance (mainly in terms of yield) of wheat genotypes is a critical requirement for successfully developing and releasing elite wheat varieties.

The article "Ascertaining yield and grain protein content stability in wheat genotypes having the Gpc-B1 gene using univariate, multivariate, and correlation analysis" was published in 2022. Journal: Front Genet.

Analysis of variance (ANOVA) is generally performed to ascertain the presence of GEI utilizing the data collected from the multi-environment trials. These measures are further used to distinguish between random (including location, replication, year, and environment) and fixed effects (such as genotypes). Nonetheless, one of ANOVA’s major flaws is its inability to distinguish genotypic variances in a non-additive base as an interaction between genotype and environment (Shahriari et al., 2018). In the literature, different statistical methods have been used to explain different parts of GEI. These methods have led to the identification of stable genotypes across locations by measuring genotypic stability. Two different approaches, including univariate (Eberhart and Ruessll’s models, Perkins and Jinks’ models, Wricke’s Ecovalnece, and Francis and Kanenberg’s model) and multivariate (AMMI and GGE biplot) stability prediction procedures, are generally utilized to better understand the phenotypic stability patterns. Pattern analysis, cluster analysis, principal component analysis (PCA), and biplot analysis are commonly utilized multivariate techniques for discovering trends of GEI (Myint et al., 2019). The biplot techniques are currently applied to diagrammatically represent the complex relationships available between the variables (genotypes, environments, and GEI) as well as to determine relatively stable genotypes throughout the environments and similarly prove the interaction structures (Shahriari et al., 2018). Singular value decomposition (SVD) and visual presentation of two-way matrices, such as the GEI statistical data, are used to develop biplots. The two most commonly used biplot analysis methods are as follows: 1) the additive main effects and multiplicative interaction (AMMI) model and 2) the genotype main effects and GE effects (GGE) model (Gauch, 2008). Furthermore, plant breeders are more interested in the above-mentioned statistical methods (AMMI and GGE) because these methods can be applied to any two-way measure, which can come from a variety of experiments. The AMMI model employs ANOVA to examine the main effects of genotypes and environments, as well as PCA to look at residual interaction features (Singh et al., 2019). In AMMI1, the PCA1 and substantial effect of the trait are represented by the abscissa line and ordinate, respectively. But AMMI2 is a graphical depiction of summarized information based on both PC1 and PC2 values, which has significant privileges as compared to regression-based statistical tools. The GGE biplot provides a more significant diagrammatical depiction as compared to AMMI model to identify genotypes conferring best performance across all the environments under study (Shrestha et al., 2021).

The article "Ascertaining yield and grain protein content stability in wheat genotypes having the Gpc-B1 gene using univariate, multivariate, and correlation analysis" was published in 2022. Journal: Front Genet.

Furthermore, as the environment in specific areas becomes more unpredictable over time, yield stability and broad adaptability are becoming increasingly important (Singh et al., 2019). In cereals, the AMMI technique was used in multi-environment experiments to characterize the most stable cultivar(s) (Sabaghnia et al., 2008; Sharifi et al., 2017). Several other studies have been successfully implemented cultivar stability analysis using both genotype and environmental assessments, as well as the GGE biplot-adopted multi-environment test, with great success (e.g., Mostafavi et al., 2011; Bishnoi and Om Perkash, 2020; Ruswandi et al., 2021). On the other hand, Gauch et al. (2008), criticized the GGE biplot structure for decomposing G + GxE, but still reported that biplots interpret G + GxE more accurately than AMMI matrices. GGE biplot analyses have widely been utilized to characterize mega-environments, examine genotype rankings, and further identify discriminativeness and representativeness in evaluated environments (Verma et al., 2015). In a multi-dimensional environment, AMMI can better identify GEI and depict it using a biplot. Both GGE and AMMI analysis models have been utilized successfully in many studies to investigate interaction patterns in multi-environment trials to discover stable genotypes of different cereals, including wheat (Singh et al., 2019; Hilmarsoon and Rio, 2021; Khan et al., 2021). The objectives for this study were to examine GEI, the performance and stability of advanced wheat genotypes, the correlation of grain yield with GPC and agronomic traits, and to ascertain the representativeness and discriminativeness abilities of the environments where wheat is grown.

The article "Ascertaining yield and grain protein content stability in wheat genotypes having the Gpc-B1 gene using univariate, multivariate, and correlation analysis" was published in 2022. Journal: Front Genet.

## Materials and methods

### Plant materials

The current research was conducted in the Department of Plant Breeding and Genetics, Punjab Agricultural University (PAU), Ludhiana, Punjab, India. For this study, a total of 13 wheat genotypes, including 9 near isogenic lines (NILs) and 4 checks, including one advanced breeding line (BWL6228), and three commercial wheat varieties (PBW761, PBW725 and HD3086), were utilized. A set of NILs was previously generated in Department of Plant Breeding and Genetics, PAU, with an aim to introgress *Gpc-B1* gene from GLUPRO into the background of a high-yielding wheat variety (PBW550). PBW550 was released by Punjab Agricultural University, Ludhiana, for cultivation under timely sown irrigated condition of north western plain zone (NWPZ), including Punjab. The variety is known for its short duration, bold, hard, and amber colored shiny grain with above average quality parameters. From this set of developed NILs, we selected the 9 most agronomically superior wheat NILs for the present study (information on pedigree of these NILs is provided in Table 1). Subsequently, the presence of Gpc-B1 in the above-mentioned NILs using the appropriate KASP marker (data not provided) was also confirmed. For the purpose of the analysis, all the NILs and checks were termed as genotypes.

**TABLE 1:** List and pedigree of the selected genotypes (nine NILs, one advanced breeding line and three released varieties) evaluated in the present study.

S. No.	Genotypes	*Gpc-B1*	Pedigree
1	BWL6228	−	BWL 2760/BWL 1879//BWL 2752/BWL 1797
2	BWL6964	+	PBW550//*Yr15*/6*Avocet/3/2*PBW550/4/GLUPRO/3*PBW568//3*PBW550
3	BWL7493	−	PBW550//*Yr15*/6*Avocet/3/2*PBW550/4/GLUPRO/3*PBW568//3*PBW550
4	BWL7495	−	PBW550//*Yr15*/6*Avocet/3/2*PBW550/4/GLUPRO/3*PBW568//3*PBW550
5	BWL7497	−	PBW550//*Yr15*/6*Avocet/3/2*PBW550/4/GLUPRO/3*PBW568//3*PBW550
6	BWL7504	+	PBW550//*Yr15*/6*Avocet/3/2*PBW550/4/GLUPRO/3*PBW568//3*PBW550
7	BWL7506	+	PBW550//*Yr15*/6*Avocet/3/2*PBW550/4/GLUPRO/3*PBW568//3*PBW550
8	BWL7508	+	PBW550//*Yr15*/6*Avocet/3/2*PBW550/4/GLUPRO/3*PBW568//3*PBW550
9	BWL7509	+	PBW550//*Yr15*/6*Avocet/3/2*PBW550/4/GLUPRO/3*PBW568//3*PBW550
10	BWL7511	+	PBW550//*Yr15*/6*Avocet/3/2*PBW550/4/GLUPRO/3*PBW568//3*PBW550
11	PBW 761	−	PBW550//*Yr15*/6*Avocet/3/2*PBW550
12	PBW725	−	PBW621//GLUPRO/3*PBW568/3/PBW621
13	HD3086	−	DBW 14/HD 2733//HUW 468

+ indicates the presence of *Gpc-B1*, gene and −indicates the absence of *Gpc-B1*, gene.

The article "Ascertaining yield and grain protein content stability in wheat genotypes having the Gpc-B1 gene using univariate, multivariate, and correlation analysis" was published in 2022. Journal: Front Genet.

Genotype 1 is an advanced breeding line, the genotypes 2–10 are near-isogenic lines, and genotypes 11–13 are released wheat varieties.

### Testing environments and crop management practices

The research trials were conducted across four locations (Ludhiana, Ballowal, Patiala, and Bathinda) of Punjab for two consecutive main crop seasons (2019–20 and 2020–21) in Punjab, India. Temperature, rainfall (Table 2) and other ecological conditions differed significantly across the environments (integration of location and time). In each environment, the experiment was conducted in a randomized block design (RBD) with three replications. Each genotype was planted in a separate plot of size 5.4 m^2^ (4.5 m long with six rows, and the distance between two rows was 20 cm). One experimental trial was sown at the wheat experimental area, wheat section, Department of Plant Breeding and Genetics, PAU, Ludhiana, and the other three were sown at the regional research stations (RRSs) of PAU located in Ballowal, Patiala, and Bathinda, respectively. All the trials were sown from November 10—November 25 in both the years 2019–20 and 2020–21. In each year, during the cropping season, weeding, irrigation, fertilizer application, and all other field management activities were applied according to the standard agronomical package recommended by PAU (https://www.pau.edu/content/ccil/pf/pp_rabi.pdf). The standard rate of fertilizer prescribed by PAU (N = 50 kg/acre, *p* = 25 kg P_2_O_5_/acre, and K = 12 kg K_2_O/acre) was applied for raising the crop. In each research location, the field was mechanically prepared in accordance with the local farmers’ interests. Furthermore, insect and disease prevention practices were implemented wherever required. Similarly, manual weeding was practiced as per requirement, and weeds were controlled with herbicide application prior to and after field preparation and also across the surrounding marginal areas of the experimental field.

**TABLE 2:** Details of environmental condition for the experimental locations (Ludhiana, Ballowal, Patiala, and Bathinda) during two consecutive years (2019–20, and 2020–21).

Pincode	Location	Latitude	Longitude	Altitude (m)	Year	Env. Condition	Nov.	Dec.	Jan.	Feb.	Mar.	Apr.
141001	Ludhiana	30˚90′10´´	75˚80′71´´	247	2019–20	Temperature	11–30°C	5–24°C	2–22°C	5–26°C	10–29°C	15–37°C
						Rainfall	35.2 mm	46.8 mm	39.8 mm	15 mm	69 mm	13.2 mm
					2020–21	Temperature	9–31°C	4–26°C	4–24°C	6–33°C	13–35°C	14–40°C
						Rainfall	16.6 mm	6 mm	11 mm	17 mm	5 mm	14.3 mm
141202	Ballowal	30˚77′09´´	75˚74′73´´	246	2019–20	Temperature	11–30°C	5–24°C	2–22°C	5–26°C	10–29°C	15–37°C
						Rainfall	16.2 mm	23.4 mm	19.5 mm	8.2 mm	25.3 mm	6.9 mm
					2020–21	Temperature	9–31°C	4–26°C	4–24°C	6–33°C	13–35°C	14–40°C
						Rainfall	6.3 mm	5 mm	8 mm	11 mm	4 mm	8.2 mm
147001	Patiala	30˚34′49´´	76.33754	280	2019–20	Temperature	11–30°C	5–24°C	2–22°C	5–26°C	10–29°C	15–37°C
						Rainfall	11.2 mm	27.1 mm	16 mm	6.7 mm	21 mm	9.9 mm
					2020–21	Temperature	9–31°C	4–26°C	4–24°C	6–33°C	13–35°C	14–40°C
						Rainfall	6 mm	5 mm	7 mm	8 mm	3 mm	11.2 mm
151005	Bathinda	30˚11′08´´	74˚56′52´´	210	2019–20	Temperature	10–32°C	2–23°C	3–22°C	5–27°C	11–30°C	14–40°C
						Rainfall	9 mm	13.2 mm	11.2 mm	4 mm	9 mm	3.2 mm
					2020–21	Temperature	8–33°C	4–36°C	2–23°C	6–36°C	14–40°C	12–43°C
						Rainfall	5 mm	7 mm	6 mm	3 mm	5 mm	2 mm

Source: https://www.timeanddate.com/weather/india/

The article "Ascertaining yield and grain protein content stability in wheat genotypes having the Gpc-B1 gene using univariate, multivariate, and correlation analysis" was published in 2022. Journal: Front Genet.

### Data collection

Data was recorded on different traits including number of days to flowering (DTF), number of days to maturity (DTM), plant height (cm; PH), number of spikelet per spike (SPS), number of grains per spike (GPS), thousand grain weight (g; TGW), grain yield (kg/plot), and grain protein content (%; GPC). These traits have an immediate and positive impact on grain yield and quality. Pre-harvest (viz., DTF, DTM, PH) and post-harvest (viz., GPS, SPS, TGW, yield and GPC) data were collected in the field, wheat quality laboratory, and molecular wheat laboratory, wheat section, Department of Plant Breeding and Genetics, PAU. Five randomly selected individual plants from each plot were considered for data recording. Data on the various traits was collected on wheat genotypes for two consecutive years (2019–20 and 2020–21) in the following manner: The DTF was recorded when 75% of the spikes emerged from boots in each plot. The DTM was recorded as the number of days from sowing to date when 75% of the spikes in plots turned yellow. PH was measured using the meter rod by placing the meter along the plant from base to tip of the ear at maturity. SPS was determined by counting the number of total spikelets on each spike. The GPS was measured by threshing the representative spikes individually and collecting, cleaning, and counting the grains manually. From harvested grains, 1000 seeds were taken from each plot, and their weight was recorded as a TGW. After threshing of each plot, the grain was weighted and considered as yield per plot. The whole grain analyzer “Infratec1241” (M/S Foss Analytical AB, Sweden) was used to measure the GPC in the grains. It is based upon the principle of near-infrared light, which is transmitted through the grains. The 200 g grain samples were scanned with a bandwidth of 7 nm in the range of 850–1050 nm, and there were 100 data points per scan.

The article "Ascertaining yield and grain protein content stability in wheat genotypes having the Gpc-B1 gene using univariate, multivariate, and correlation analysis" was published in 2022. Journal: Front Genet.

### Statistical analysis

Using different packages of R software version 4.0.5, the data on different quantitative traits was subjected to a combined ANOVA to determine whether there was any variation among all the variables considered during the current study. Environments were considered random variables, while genotypes were treated as fixed variables. The Pearson correlation along with the pattern were prepared using “corroplot” package of R software, using the following model given as:

$rG=\frac{cov\;\left(A,\;B\right)}{\sqrt{var\left(A\right)\;.\;var\left(B\right)}}$ Where *cov* (*A*, *B*) indicates the covariance present between independent and dependent traits, and *var* (*A*)*,* and also *var* (*B*) shows the genetic difference of independent and dependent trait (Sandhu et al., 2021a). For further analysis, we only utilized the data on GPC and grain yield, as they are both considered the critical traits in terms of total wheat production and nutritional security. To study the GEI, first, the univariate stability analysis of the genotypes under study was conducted using regression analysis based on the six different univariate stability measures: Eberhart and Russell’s (1966) regression coefficient (*bi*) and deviation from regression (*S* ^*2*^ *di*) determine the performance of a genotype across different environments (Changizi et al., 2014). The Eberhart and Russell’s (1966) stability model is given as: Y_ij_ = μ_i_ + β_i_I_j_ + δ_ij_, where the Y_ij_ indicates the evaluation of *i*th (i = 1, 2, 3,……, x) genotype across the *j*th (1, 2, 3,……, *n*) environment, μ_i_ is the genotype mean, β_i_ indicates the regression coefficient, δ_ij_ shows the deviation from the regression coefficient, and I_j_ is the environmental index identified by subtracting the total mean from each environmental mean (Francis and Kanenberg’s 1978). coefficient of variability, which shows the CV% of every individual genotype as a stability parameter. Perkins and Jinks (1968), regression coefficient (*Bi*) and deviation from regression (*DJi*), using the following model as represented here: Y_ij_ = μ + AG_i_ + AE_j_ + GE_ij_ + ER_ij_, where Y_ij_ is the performance of *i*th genotype in the *j*th environment, μ represents general mean over all the genotypes and environments, AG_i_ is additive genetic portion of *i*th genotype, AE_j_ shows the additive environmental portion of *j*th environment, GE_ij_ represents the GEI of *i*th genotype in *j*th environment, and ER_ij_ is the experimental error for *i*th genotype in the *j*th environment. Furthermore, the Wricke’s (1962) ecovalence (*Wi*), which indicates the GEI for individual genotypes across all the tested environments. Ecovalence, is used identify the effective contribution of the genotypes to the overall GEI, and calculated through the given formula: $\bar{\sum }\left[xij-\frac{Xi.}{q}-\frac{X.i}{p}-\frac{X..}{pq}\right]$ , where *X*_*ij*_ is the evaluation of *i*th genotypes in *j*th environment, *X*_*i.*_ = total sum of *i*th genotype across all the studied environments, *X*_*. i*_ = total sum of *i*th environment for all the studied genotypes, q is all the environments, and *p* shows all the genotypes. Then the multivariate approaches for stability analysis were conducted according to AMMI and GGE biplot using different statistical packages available in R studio. The “metan” package of R studio was applied for AMMI analysis, while the GGEBiplotGUI package was employed for GGE biplot based analysis. In the AMMI model, the ANOVA and PCA are merged together into an individual statistical package. Therefore, GEI is subjected to PCA analysis only when primary verification has already been completed using ANOVA (Neisse et al., 2018). The equation for AMMI model is given as below: Y_ge_ = μ + α_g_ + β_e_ + Σ_n_λ_n_γ_gn_δ_en_ + ρ_ge_, where in case of the additive factors, Y_ge_ is showing the grain yield for a particular (g) genotype in an (e) environment, where μ stand for grand mean, α_g_ indicates deviation of genotype from the mean, β_e_ is deviation of environment from the mean, λ_n_ stands for singular value of n component, γ_gn_ indicates the value of eigenvector for genotype (g) and δ_en_ is the value of eigenvector for e and ρ_ge;_ which is known as residual (Rad et al., 2013). Furthermore, the equation for GGE biplot model is represented as: P_ij_ = (y_ij_—μ—δ_j_)/λ_j_ = (β_i_ + ϵ_ij_)/λ_j_, where P_ij_ is the matrix for genotype i and environment j, μ represents the grand mean, δ_j_ is the column (environment) main effect, λ_j_ is an evaluating factor, β_i_ is the row (genotype) main effect, and ϵ_ij_ represents GEI, and y_ij_ is G and E two-way table (Yan and Tinker, 2006). Also, the GGE biplot involves a group of bioplot-based platforms for the interpretation of interactions present between the genotype and the environment. In general, in both GGE biplot and AMMI, the graphical images are used to answer the critical queries about G x E evaluation on a visual basis (Pour-Aboughadareh et al., 2022). In addition, in both the biplot analyses, the results are further interpreted based on the criteria mentioned by Khan et al. (2021).

The article "Ascertaining yield and grain protein content stability in wheat genotypes having the Gpc-B1 gene using univariate, multivariate, and correlation analysis" was published in 2022. Journal: Front Genet.

## Results

### Correlation

Figure 1 provides information regarding the correlation values and patterns among the different traits in question with a particular focus on yield and GPC across all the environments. Yield was observed to have a highly significant negative correlation with GPC (−0.52), while conferring a highly significant positive correlation with TGW (0.66), DTM (0.57). GPC had a highly significant negative correlation with DTF (−0.55), PH (−0.57), DTM (-0.83), TGW (−0.75), and yield (−0.52).

**FIGURE 1:** Pattern of correlation and level of significance observed among different traits across all the environments in 13 bread wheat genotypes. DTF, Number of days to flowering; PH, Plant height; SPS, Number of spikelets per spike; GPS, Number of grain per spike; DTM, Number of days to maturity; TGW, 1000-grain weight; GPC, Grain protein content.

### Pooled analysis of variance for yield, grain protein content and their related traits

The pooled ANOVA was performed to unravel the main effect and determine the interaction present within and among the sources of variations that are analyzed during the present study. The pooled ANOVA concerning all the eight traits is presented in Table 3. The variance due to genotype (G), location (L), year (Y), G × Y, G × L, and G × Y × L for all the eight traits was highly significant, either at 0.001% or at 0.01% level of significance. A high level of variability was observed in wheat genotypes for key traits related to yield and GPC.

**TABLE 3:** Combined analysis of variances for grain protein content, yield and key yield-related traits of 13 bread wheat genotypes across eight environments.

S.V		DTF		PH		SPS		GPS	
	DF	SS	MS	SS	MS	SS	MS	SS	MS
Genotype	12	1497	124.8***	2944	245.4***	53.13	4.43***	832	69***
Location	3	5006	1668.8***	3293	1097.6***	178.47	59.49***	10425	3475***
Year	1	15	14.48***	23	23.4***	29.54	29.54***	907	907***
G × Y	12	43	3.6***	172	14.3***	25.71	2.14***	178	15**
G × L	36	230	6.4***	1274	35.4***	68.70	1.91***	1468	41***
Y × L	3	49	16.3***	221	73.7***	72.90	24.30***	1713	571***
G × Y × L	36	263	7.3***	588	16.3***	91.76	2.55***	540	15***
**S.V**		**DTM**		**Yield**		**TGW**		**GPC**	
	**DF**	**SS**	**MS**	**SS**	**MS**	**SS**	**MS**	**SS**	**MS**
Genotype	12	653	54.5***	11.03	0.920***	978	81.5***	268.50	22.37***
Location	3	4216	1405.2***	93.27	31.090***	4059	1353***	130.11	43.37***
Year	1	33	32.7***	0.06	0.064^ns^	2	1.9^ns^	12.87	12.87***
G × Y	12	11	0.9^ns^	9.74	0.812***	189	15.8***	16.88	1.41***
G × L	36	441	12.3***	94.47	2.624***	723	20.1***	46.41	1.29***
Y × L	3	340	113.2***	16.37	5.458***	54	18.1***	7.57	2.52***
G × Y × L	36	147	4.1***	25.66	0.713***	437	12.1***	27.69	0.77***

** , 0.01% level of significance.

***, 0.001% level of significance.

ns, Non-significant; DF, Degrees of freedom; SS, sum of squares; MS, Mean square,;S.V, Source of variances; G × Y, Genotype × Year; G × L, Genotype × Location; Y × L, Year × Location; G × Y × L, Genotype × Year × Location; DTF, Number of days to flowering; PH, Plant height; DTM, Number of days to maturity; SPS, Number of spikeletes per spike; GPS, Number of grain per spike; TGW, 1000-grian weight, and GPC, Grain protein content.

The article "Ascertaining yield and grain protein content stability in wheat genotypes having the Gpc-B1 gene using univariate, multivariate, and correlation analysis" was published in 2022. Journal: Front Genet.

### Univariate analyses

The data for different regression stability analyses is presented in Table 4 (concerning GPC, and yield) and Supplementary Table S1 (concerning DTF, DTM, SPS, GPS, TGW, and PH). In this study, we focused specially on yield and GPC. For yield, based on the Eberhart and Russell (1966) model, the deviations from the regression (S2di) indicated that, BWL7495, BWL7509, and PBW761 are stable genotypes and, accordingly, the coefficient of regression (bi) showed that they are adaptable, particularly to unfavorable environments (bi = 0.7491 for BWL7495, *bi* = 0.5863 for BWL7509, and bi = 0.607 for PBW761), but BWL7511 showed adaptability specific to high-yielding environments (bi = 1.1432). The genotypes, BWL7495, BWL7509, PBW725, HD3086, and PBW761 are categorized in the class of stable and high-yielding genotypes, which are adapted particularly to low-performing environments. These genotypes are grouped in this class based on their regression values, which is lower than one. Based on mean grain yield, the BWL7497, BWL7509, PBW761, and PBW725 showed the highest yield and, therefore, were preferred over other genotypes. These genotypes are grouped based on their mean in the high-yielding class. Based on Perkins and Jinks regression analysis, the genotype BWL6964 had a positive coefficient, but the genotypes, BWL7495, BWL7509, and PBW761 had negative coefficient values. Consequently, BWL6964 was observed to be stable due to its highest regression value and adapted specifically to high-yielding environments. Furthermore, the variation in the mean value for yield could be described by the respective responses of genotypes across environments. The regression value close to 1 confirms that genotypes perform in a stable manner across all the environments. The genotypes BWL7508 (bi = 1.15, CV = 16.6%, Bi = 0.15, mean = 2.83 kg/plot; Table 4, and Supplementary Table S2) and BWL7511 (bi = 1.14, CV = 14.87%, Bi = 0.14, mean = 2.81 kg/plot; Table 4, and Supplementary Table S2) were selected as the most stable and producing high yield.

The article "Ascertaining yield and grain protein content stability in wheat genotypes having the Gpc-B1 gene using univariate, multivariate, and correlation analysis" was published in 2022. Journal: Front Genet.

**TABLE 4:** Six univariate stability parameters and standard deviation for (**A**) yield and (**B**) GPC of 13 wheat genotypes across four locations (Ludhiana, Ballowal, Patiala, and Bathinda) of Punjab in two consecutive years 2019–20, and 2020–21. (A) Yield and (B) Grain protein content (GPC).

Genotypes		Francis and kanenberg	Eberhart and russell		Perkins and jinks		Wricke’s ecovalence
	*Sd*	CV (%)	*bi*	*S* ^*2*^ *di*	*Bi*	*DJi*	*Wi*
BWL6228	1.1151	22.1484	0.859	1.0742	−0.141	1.1049	6.6854
BWL6964	1.2438	23.5916	1.712	0.4009	0.712	0.4316	4.0149
BWL7493	1.1008	21.2189	1.1536	0.7595	0.1536	0.7902	4.8076
BWL7495	0.5786	11.9541	0.7491	0.097	−0.2509	0.1277	0.9433
BWL7497	1.0779	20.1607	1.3935	0.415	0.3935	0.4457	3.1097
BWL7504	1.0069	20.0641	1.3718	0.2704	0.3718	0.3011	2.1953
BWL7506	1.224	23.878	1.2797	0.9499	0.2797	0.9806	6.1036
BWL7508	0.8715	16.6017	1.1553	0.2299	0.1553	0.2606	1.6313
BWL7509	0.487	9.2235	0.5863	0.085	-0.4137	0.1157	1.1753
BWL7511	0.7742	14.8713	1.1432	0.0562	0.1432	0.0869	0.5791
HD3086	0.7772	14.9953	0.1619	0.6618	-0.8381	0.6925	6.1301
PBW725	0.9882	17.4926	0.8277	0.7876	-0.1723	0.8183	4.993
PBW761	0.4629	8.6203	0.607	0.0467	-0.393	0.0773	0.8983

Genotypes		Francis and kanenberg	Eberhart and russell		Perkins and jinks		Wricke’s ecovalence
	*Sd*	CV (%)	*bi*	*S* ^*2*^ *di*	*Bi*	*DJi*	*Wi*
BWL6228	0.7676	6.0004	0.8626	0.1807	−0.1374	0.2086	1.3248
BWL6964	0.8503	6.2098	0.996	0.1774	−0.004	0.2053	1.232
BWL7493	1.375	10.2205	1.6906	0.3388	0.6906	0.3667	4.0414
BWL7495	1.3797	10.2976	1.7058	0.3207	0.7058	0.3486	4.0147
BWL7497	0.8149	6.2211	0.9703	0.1411	−0.0297	0.169	1.0176
BWL7504	1.0129	7.3816	1.2902	0.0979	0.2902	0.1258	1.0801
BWL7506	0.568	4.2377	0.2713	0.3011	−0.7287	0.329	4.0242
BWL7508	0.9113	6.5333	1.0658	0.2101	0.0658	0.238	1.4447
BWL7509	1.034	7.5539	1.3295	0.0822	0.3295	0.1101	1.0796
BWL7511	0.9777	7.1727	1.2088	0.147	0.2088	0.1749	1.218
HD3086	0.7704	6.6667	0.8192	0.2329	−0.1808	0.2608	1.6908
PBW725	0.4421	3.9949	0.1342	0.1886	−0.8658	0.2165	4.1924
PBW761	0.8594	7.4214	0.6556	0.5571	−0.3444	0.585	3.9679

*Sd*, Standard deviation; *CV*, coefficient of variation; *bi*, Regression coefficient of Eberhart and Russell; *S* ^*2*^ *di*, Deviation form regression of Eberhart and Russel; *Bi*, Regression coefficient of Perkins and Jinks; *DJi*, Deviation from regression of Perkins and Jinks; *Wi*, Wrick’s equivalence.

In the case of GPC, the (*S* ^*2*^ *di*) showed that BWL6228, BWL6964, PBW761, and PBW725 are the genotypes with high stability, and based on (*bi*) they are considered to have specific adaptation to low-yielding environments (*bi* = 0.862 for BWL6228, *bi* = 0.996 for BWL6964, *bi* = 0.65 for PBW761, and *bi* = 0.134 for PBW725), but BWL7511 is observed to be particularly adapted to high-yielding environments (*bi* = 1.2088). The genotypes BWL6228, BWL6964, BWL7497, BWL7506, PBW761, PBW725, and HD3086 are grouped as the high-GPC and stable genotypes and showed specific adaptability to unfavorable environments because they had regression value of less than 1 (*bi < 1*). On the other hand, BWL6964, BWL7504, BWL7508, and BWL7509 had GPC greater than the average mean, and therefore, they could be more desirable than other genotypes. They are considered as high-GPC genotypes based on their GPC mean. According to Perkins and Jinks’ regression model, the genotype BWL7495 showed a positive regression value, but the genotypes BWL6228, BWL6964, BWL7511, PBW761, and PBW725 showed negative regression values. Therefore, BWL7495 was recorded as a stable genotype because of its highest coefficient value (*Bi* = 0.705) and therefore, it was adapted particularly to favorable environments. The regression value near to 1 indicates that genotypes perform at a stable level across all the environments. The genotypes BWL7508 (*bi* = 1.06, *CV* = 6.53%, *Bi* = 0.06, mean = 13.94%), and BWL7511 (*bi* = 1.20, *CV* = 7.17, *Bi* = 0.20, mean = 13.63%) were identified as the most stable genotypes and had high GPC.

The article "Ascertaining yield and grain protein content stability in wheat genotypes having the Gpc-B1 gene using univariate, multivariate, and correlation analysis" was published in 2022. Journal: Front Genet.

### Additive main effects and multiplicative interaction based analysis of variance for yield, grain protein content and their related traits

The AMMI based ANOVA involving all the eight traits evaluated in the present study is given in Table 5. The results revealed that the DTF, PH, SPS, GPS, TGW, yield, GPC, and DTM are significantly influenced at a 0.001% level of significance by G, E, and GEI. The environment explained more than 50% of the total variation for all the traits except yield, GPC, and PH. For instance, the proportion of total variation contributed by G, E, and GEI for grain yield was 43.78, 4.4, and 51.83%, respectively. In the case of GPC, genotype, GEI, and E contribution explained 52.64, 17.84, and 29.52% of the total phenotypic variation, respectively. The genotype contributed less than 35% of the total observed variation for all the traits except GPC.

**TABLE 5:** AMMI-based ANOVA for yield, GPC and their related traits of 13 bread wheat genotypes across four locations (Ludhiana, Ballowal, Patiala, and Bathinda) of Punjab in two consecutive years 2019–20, and 2020–21.

		DTF			PH		
	DF	SS	MS	% Explained	SS	MS	% Explained
Environment	7	5069.99	724.28***	71.37	3537.61	505.37***	41.54
Genotype	12	1497.07	124.76***	21.08	2944.48	245.37***	34.58
G × E	84	536.263	6.385***	7.55	2033.65	24.210***	23.88
PC1	18	222.982	12.39***	41.58	1206.63	67.035***	59.33
PC2	16	122.378	7.65***	22.82	432.88	27.055***	21.29
		**SPS**			**GPS**		
	**DF**	**SS**	**MS**	**% explained**	**SS**	**MS**	**% explained**
Environment	7	280.91	40.13***	54	13045.22	1863.60***	81.21
Genotype	12	53.135	4.43***	10.21	832.45	69.37***	5.18
G × E	84	186.17	2.22***	35.79	2185.72	26.02***	13.61
PC1	18	67.120	3.73***	36.05	1147.88	65.27***	53.75
PC2	16	37.200	2.33***	19.98	409.29	25.58***	18.73
		**DTM**			**Yield**		
	**DF**	**SS**	**MS**	**% explained**	**SS**	**MS**	**% explained**
Environment	7	4587.84	655.41***	78.56	109.64	15.66***	43.78
Genotype	12	652.52	54.38***	11.17	11.03	0.92***	4.40
G × E	84	599.39	7.14***	10.26	129.80	1.55***	51.83
PC1	18	347.63	19.31***	58	69.77	3.88***	53.75
PC2	16	118.21	7.39***	19.72	24.91	1.56***	19.19
		**TGW**			**GPC**		
	**DF**	**SS**	**MS**	**% explained**	**SS**	**MS**	**% explained**
Environment	7	4115.20	587.88***	63.87	150.55	21.51***	29.52
Genotype	12	977.83	81.49***	15.18	268.51	22.38***	52.64
G × E	84	1350.09	16.07***	20.95	90.98	1.08***	17.84
IPC1	18	571.13	31.73***	42.30	46.39	2.58***	50.99
IPC2	16	390.78	24.42***	28.94	16.93	1.06***	18.61

*** , 0.001% level of significance.

The article "Ascertaining yield and grain protein content stability in wheat genotypes having the Gpc-B1 gene using univariate, multivariate, and correlation analysis" was published in 2022. Journal: Front Genet.

DF, Degree of freedom; SS, Sum of square; MS, Mean square; G × E, Genotype × Environment; DTF, Number of days to flowering; PH, Plant height; DTM, Number of days to maturity; SPS, Number of spikelets per spike; GPS, Number of grain per spike; TGW, 1000-grian weight, and GPC, Grain protein content.

### Genotype × environment interaction based on additive main effects and multiplicative interaction model

It allowed us the opportunity to look at the biplot graph when it was chosen to apply AMMI-based analysis to examine both the adaptability and stability of genotypes. The predicted variation among and within the main effects of either G or E, as well as the multiplicative interaction of the GEI, are efficiently used to explain the biplot graphs. In a biplot graph, the main effects (mean performance of tested genotypes) are displayed by the abscissa, while the possible interaction among the axes (IPCA1 and IPCA2) is represented by the ordinate (Oliveira et al., 2014). Thus, the higher PCA1, the higher the proportion of GEI and, consequently, the lower stability of lines under study or vice versa. By keeping this in view, a high-yielding genotype with an IPCA1 score adjacent to the zero line is preferred. On the other hand, poor stability is related to low performance of the trait, hence this genotype is not preferred. Different responses of environment to genotypic stability for the tested genotypes were observed in the present study. Figure 2 represents the AMMI1 based analysis of 13 genotypes and 8 environments for yield, and GPC. Based on PCA1 value, the ENV4 is determined as the major player to the stability performance of genotypes in case of yield and GPC. On the other hand, BWL7495 and PBW761 for yield (Figure 2A), BWL7504 for GPC (Figure 2B) secured an IPCA1 value of close to zero suggesting minor environmental effect on these genotypes.

The article "Ascertaining yield and grain protein content stability in wheat genotypes having the Gpc-B1 gene using univariate, multivariate, and correlation analysis" was published in 2022. Journal: Front Genet.

**FIGURE 2:** The “AMMI1” graphs displays the main effect and IPC1 effect values describing relationship among examined genotype and environment of 13 bread wheat genotypes across four locations (Ludhiana, Ballowal, Patiala, and Bathinda) of Punjab in two consecutive years (2019–20, and 2020–21) for **(A)** yield (kg/plot) and **(B)** GPC (%). (ENV1, and ENV5 = Ludhiana; ENV2, and ENV6 = Ballowal; ENV3, and ENV7 = Patiala; ENV4, and ENV8 = Bathinda).

For AMMI2, the biplot graph representing the environment and genotype stability performance of yield and GPC is provided in Figure 3. In case of AMMI2, the genotypes and environments with lower IPCA1 and IPCA2 value that are securing a closer position to the origin are considered as the most stable ones which explained lower interaction between environment and genotype. In the present study, the BWL7508, BWL7509, and BWL7511 for instance, considered as the most stable wheat genotypes in terms of yield (Figure 3A), based on the their positions near to the origin. In case of GPC, the BWL7497, BWL7504, and BWL7511 are suggested as the most stable ones (Figure 3B). On the other hand, ENV2 and ENV4 secured positions near to origin and considered the most stable environments for all the genotypes in terms of yield and GPC, respectively.

**FIGURE 3:** The “AMMI2” graphs displays both the axes of interaction (IPCA1 and IPCA2) values for genotype effect and genotype by environment interaction effect of 13 bread wheat genotypes across four locations (Ludhiana, Ballowal, Patiala, and Bathinda) of Punjab in two consecutive years (2019–20 and 2020–21) for **(A)** yield (kg/plot) and **(B)** GPC (%). (ENV1, and ENV5 = Ludhiana; ENV2, and ENV6 = Ballowal; ENV3, and ENV7 = Patiala; ENV4, and ENV8 = Bathinda).

### GGE biplot based evaluation of genotype × environment interaction

The predominant control of the genotype and its interaction with the environment is considered the fundamental origin of variations whenever, evaluating the genotypes across the multi-location trials. The three important indicators which could be determined by biplot are considered to be capable of defining the GEI are as follows: 1) the “which-won-where” graph, which is an efficient pattern to display the principle of GEI; 2) the stability vs. genotype mean performance across different environments tested in the study; and 3) the representativeness and discriminating abilities of the tested environments.

The article "Ascertaining yield and grain protein content stability in wheat genotypes having the Gpc-B1 gene using univariate, multivariate, and correlation analysis" was published in 2022. Journal: Front Genet.

### “Which-won-where” approach

The polygon-view of a GGE biplot analysis illustrates the which-won-where structure of a multi-environment experiment, which is consequently the most efficient and simplest manner of characterizing the genotype and its further interaction with the environment. Figures 4A,B describe the which-won-where structure of biplot analysis for yield and GPC of 13 wheat genotypes distributed over all the 6 sectors/sections, while the 8 tested environments are distributed over 4 sectors for yield and 3 sectors for GPC. In terms of yield, sector 1 consists of ENV1 and ENV5 along with wheat genotypes BWL7497, BWL7506, and BWL7511; sector 2 contains ENV2 and ENV6 with BWL6964 and BWL7493; sector 5 carries ENV4 and ENV7 with BWL7508 and PBW726; and sector 6 consists of ENV3 and ENV8 with BWL6228 (Figure 4A). The genotypes are more suitable and confer a high level of performance and stability in the environment within the same sector. The elite variety PBW725 is observed to be the most away from the biplot origin and also the polygon vertex line, indicating that PBW725 confers a high level of adaptability and yield performance specific to ENV4 and ENV7, but shows poor stability across all other tested environments. In case of GPC, sector 2 carries ENV1 with BWL7509, sector 3 contains ENV2, ENV3, ENV4, ENV5, ENV6, and ENV7 along with wheat genotype BWL7511, and sector 4 carries ENV8 with BWL6964, BWL7504, BWL7506, and, BWL7508 confirming that these genotypes are more suitable and confer a high level of performance and stability in the environment within the same sector, but less stable and poor performance across environments in different sectors. In case of GPC, the genotype BWL7506 showed the longest distance from the biplot center and the polygon vertex line which indicates that BWL7506 confers high stability and has good performance as well as good adaptation specifically to ENV8, but poor adaptation to other environments (Figure 4B). Furthermore, the genotype with close contact to the vertex line of the polygon in a section where the environments are also observed in that section showed that the observed genotype conferred higher performance and adaptation in that particular environment. In case of GPC, for instance, the genotype BWL7497 was in close contact with vertex line, therefore, had high-GPC performance and adaptability specifically to ENV1. A genotype connected to a polygon vertex line where no environment is observed indicates that the genotype is providing lower yield or performance over all the environments. Even more, the genotypes inside the polygon are less affected by the environment than the genotypes at the corners are.

The article "Ascertaining yield and grain protein content stability in wheat genotypes having the Gpc-B1 gene using univariate, multivariate, and correlation analysis" was published in 2022. Journal: Front Genet.

**FIGURE 4:** The polygon view of “Which-won-where” model of GGE biplot representing the performance of 13 bread wheat genotypes and their interactions with environment across four locations (Ludhiana, Ballowal, Patiala, and Bathinda) of Punjab in two consecutive years (2019–20, and 2020–21) based on **(A)** yield (kg/plot and **(B)** GPC (%). (ENV1, and ENV5 = Ludhiana; ENV2, and ENV6 = Ballowal; ENV3, and ENV7 = Patiala; ENV4, and ENV8 = Bathinda).

### Means versus stability model of GGE biplot and evaluation of wheat genotypes

After the which–won–where model of GGE biplot recommended the dominating wheat genotypes under certain environments, it became essential to evaluate the average stability and performance of all wheat NILs before making a selection choice. The performance and stability of the genotypes are graphically represented by the GGE biplot using average environmental coordinates (AEC). If single value portioning (SVP) is equal to 1, the AEC line crosses through the origin of the biplot. This biplot graph is made up of two lines which are perpendicular to each other: 1) the AEC abscissa and 2) the AEC ordinate. The arrowhead in Figures 5A,B represents the AEC, which is the average of the first and second PCA values of the evaluated environments. The AEC abscissa is the line crossing through the origin and arrowhead, pointing to higher mean performance of certain traits, and its length indicates the magnitude of the genotype’s performance for a particular trait, which is either above or below the average performance of the genotype with respect to the right or left side of the origin point, respectively. The ordinate is the line perpendicular to the abscissa at the origin point, and its length determines the GE interaction associated with the genotype, where a longer ordinate is associated with greater variability and poor stability.

**FIGURE 5:** The “mean versus stability” model describing the interaction effect of 13 bread wheat genotypes evaluated across four locations (Ludhiana, Ballowal, Patiala, and Bathinda) of Punjab in two consecutive years (2019–20, and 2020–21) for **(A)** yield (kg/plot) and **(B)** GPC (%). (ENV1, and ENV5 = Ludhiana; ENV2, and ENV6 = Ballowal; ENV3, and ENV7 = Patiala; ENV4, and ENV8 = Bathinda).

Figure 5A indicates that the wheat genotypes BWL7497, BWL7508, and BWL7511 have above-average yield and greater stability, while BWL6228, BWL7506, and PBW725 also have above-average yield, but show poor stability. On the other hand, genotypes BWL7495, BWL7504, BWL7509, and BPW761 are stable but show yield below the average and BWL6964, BWL7493 and HD3086 have yield below-average and show less stability. The Figure 5B shows that the.

The article "Ascertaining yield and grain protein content stability in wheat genotypes having the Gpc-B1 gene using univariate, multivariate, and correlation analysis" was published in 2022. Journal: Front Genet.

BWL6964, BWL7497, BWL7504, BWL7506, BWL7508, BWL7509, and BWL7511 have above-average GPC and higher stability whereas BWL7493, and BWL7495 also have above-average GPC, but show less stability. Furthermore, the BWL6228, PBW761, PBW725, and HD3086 have GPC below-average and show more stability. Based on mean versus stability model, ideal genotypes line on the arrowhead, conferring the best performance and maximum stability while the distance between arrowhead and other genotypes determines their specific trait potential. Figures 5A,B indicate that BWL7508, and BWL7511 are the most desirable genotypes for yield and GPC, respectively, which are greatly close to the arrowhead, followed by BWL7497 for yield and BWL7504 for GPC.

### Ranking the ideal wheat genotypes

The arrowhead contains the best performing genotypes, but it is not always possible to be the ideal one. Two coordinate axes are sketched to rank the genotypes (Figures 6A,B): a straight line connecting the arrowhead with the origin of the graph (first axis) and a line exactly perpendicular to the first axis at the origin (second axis). The genotypes may then be ranked based on involvement in the circles and position located away from the arrowhead in the ordinate by viewing circles anywhere along the arrowhead. Using the ranking graph of biplot, the best and ideal genotype could be detected. The PBW725 variety is close to the arrowhead, which is considered the ideal genotype for grain yield (Figure 6A), followed by BWL7506 and so on. In the case of GPC (Figure 6B), BWL7511 is noted as the best genotype due to its closeness to the arrowhead, followed by BWL7509 and BWL7504. If we rank all the genotypes for yield based on biplot ranking decisions, it would be as follows: PBW725 > BWL7506 > BWL7508 > BWL7511 > BWL7497 > BWL6228 > BWL7509 > PBW761 > BWL6964 > BWL7493 > BWL7504 > HD3086 > BWL7495 (Table 6). Furthermore, the ranking of genotypes for yield and GPC based on biplot decision is consistent with the average performance of the genotypes for these two and other concerning traits over all the 8 environments (Supplementary Table S2).

**FIGURE 6:** The “ranking genotypes” model of biplot assess other genotypes against the ideal genotype conferring genotype interaction and GEI for 13 bread wheat genotypes evaluated across four locations (Ludhiana, Ballowal, Patiala, and Bathinda) of Punjab in two consecutive years (2019–20, and 2020–21) for **(A)** yield (kg/plot), and **(B)** GPC (%). (ENV1, and ENV5 = Ludhiana; ENV2, and ENV6 = Ballowal; ENV3, and ENV7 = Patiala; ENV4, and ENV8 = Bathinda).

The article "Ascertaining yield and grain protein content stability in wheat genotypes having the Gpc-B1 gene using univariate, multivariate, and correlation analysis" was published in 2022. Journal: Front Genet.

**TABLE 6:** Ranking of 13 bread wheat genotypes based on yield and GPC mean and biplot decision.

Rank	Mean yield based ranking	Biplot based ranking	Rank	Mean GPC based ranking	Biplot based ranking
1	PBW725	PBW725	1	BWL7508	BWL7511
2	PBW761	BWL7506	2	BWL7504	BWL7509
3	BWL7497	BWL7508	3	BWL6964	BWL7504
4	BWL7509	BWL7511	4	BWL7509	BWL6964
5	BWL6964	BWL7497	5	BWL7511	BWL7508
6	BWL7508	BWL6228	6	BWL7493	BWL7497
7	BWL7511	BWL7509	7	BWL7495	BWL6228
8	BWL7493	PBW761	8	BWL7506	BWL7493
9	HD3086	BWL6964	9	BWL7497	BWL7495
10	BWL7506	BWL7493	10	BWL6228	BWL7506
11	BWL6228	BWL7504	11	PBW761	PBW761
12	BWL7504	HD3086	12	HD3086	HD3086
13	BWL7495	BWL7495	13	PBW725	PBW725

GPC, grain protein content.

### Discriminativeness vs. representativeness of the environments

Identifying the ideal environment for testing of genotypes is more challenging for a successful breeding project aimed to select the best genotypes. Discriminativeness (an environment’s capacity to discriminate among the genotypes) and representativeness (an environment’s potential to represent all other environments evaluated) are two characteristics that indicate how perfect the tested environments are. The Figures 7A,B describes the “descriminitiveness vs. representativeness” model of biplot. The GGE biplot tests discriminativeness using the environmental vectors; the longer the environment vector, the larger the standard deviation within the environment, suggesting more discriminative ability. The selection of better genotypes is ideal in an environment with a long vector that makes a narrower angle with the AEC abscissa line. Consequently as illustrated in Figures 7A,B, ENV1 for yield and ENV3 for GPC have relatively longer vectors and narrower angles with AEC abscissa lines indicating that these environments have a better discriminating and representing capacities for yield and GPC. However, the average of grain yield and GPC were higher in ENV1 and ENV5 as compared to other environments (Supplementary Tables S3, S4). The cosine of the angle between the AEC line, and the environment vector is almost equal to the correlation coefficient between the mean performance of genotype over the environment and the genotype values in that environment. The narrower the angle between the AEC line and the environment vector (used to test the genotype), the better the environment in comparison to those that confer larger angles. The direction of the AEC abscissa line is shown by an arrow, whereas the environment mean is indicated by a tiny circle, and the length of the test environment vector reflects the discriminating accuracy level. The length of each environment vector indicates how good (discriminating capacity) it is for distinguishing genotypes in the environment.

The article "Ascertaining yield and grain protein content stability in wheat genotypes having the Gpc-B1 gene using univariate, multivariate, and correlation analysis" was published in 2022. Journal: Front Genet.

**FIGURE 7:** The “Discrimitiveness vs. Representativeness” model of biplot evaluate the genotypes anianst the ideal genotypes conferring genotype interaction and GEI for 13 bread wheat genotypes across four locations (Ludhiana, Ballowal, Patiala, and Bathinda) of Punjab in two consecutive years (2019–20, and 2020–21) for **(A)** yield (kg/plot) and **(B)** GPC (%). (ENV1, and ENV5 = Ludhiana; ENV2, and ENV6 = Ballowal; ENV3, and ENV7 = Patiala; ENV4, and ENV8 = Bathinda).

## Discussion

India is considered one of the major countries in terms of wheat production and consumption in the world. In the present study, the AMMI and pooled-based analysis of variance showed a high and significant amount of variation among 13 wheat genotypes based on eight different traits. The high level of genetic variation, which is significantly observed in the present as well as in previously published studies, using near-isogenic lines confirmed the availability of a golden opportunity to employ the near-isogenic population for wheat improvement programmes with a special focus on GPC and yield (Bányai et al., 2017; Kokhmetova et al., 2017). In this study, we particularly focused on yield and GPC for the following reasons: 1) wheat grain yield is very important since it is a stable source of food for the world’s population 2) GPC is an important determinant of food quality 3) combining higher grain yield and higher GPC in an individual wheat variety is considered as an important determinant of food and nutritional security in the world.

The yield had a strong positive correlation with 1000-grian weight (0.66). This finding is consistent with results previously reported in wheat (Mecha et al., 2017; Baye et al., 2020). The positive association of yield with 1000-grian weight suggests that it could be possible to effectively select for both the traits concurrently. Yield also showed a positive correlation with SPS (0.33), DTF (0.45), PH (0.13), and DTM (0.57). Ojha et al. (2018) reported a positive correlation between yield and plant height. A similar positive correlation between yield and spikelet per spike and the number of days to maturity was reported by Dutamo et al. (2015). Similarly, the positive correlation between yield and the number of DTF was previously reported in wheat (Gelalcha and Hanchinal, 2013). On the other hand, the significantly negative correlation between yield and GPC is in agreement with the results previously reported by some other studies (Brevis and Dubcovsky, 2010; Blanco et al., 2012). This is mostly due to a shorter grain filling period and early senescence which comes as a linked trait when introgressing *Gpc-B1* gene.

The article "Ascertaining yield and grain protein content stability in wheat genotypes having the Gpc-B1 gene using univariate, multivariate, and correlation analysis" was published in 2022. Journal: Front Genet.

In comparison to the effects of environment (29.52%) and GEI (17.84%), the effect of genotype (52.64%) highly contributed to the total variation in GPC. As a result, the genotypic component of variation explained a significant portion of the total variation for the GPC, implying that genotypes differed more than environments. However, for the remaining traits except yield, the contribution of environmental effects was higher than the effect of both the genotype and GEI to the total variances for DTF (71.37%), PH (41.54%), SPS (54%), GPS (81.21%), DTM (78.56%), and TGW (63.87%). The effect of GEI (51.83%) was higher than the effect of both the environment (43.78%) and genotype (4.4%) for yield. The greater contribution of GEI and environment to the total variation in grain yield was also observed in several earlier studies in wheat (e.g., Amare et al., 2015; Verma et al., 2015; Singh et al., 2019) and in some other crops (e.g., Rakshit et al., 2012; Mukuze et al., 2020). The highly significant contribution of the GEI effect to the total differences in yield indicates that the response of various wheat genotypes to variation in environmental factors was entirely different, implying that selection of environment-specific genotypes is required. Furthermore, the greater contribution of GEI to variation in yield over genotype suggests that there may be some different mega-environments available across the examined environments (Enyew et al., 2021). On the other hand, much larger environmental effect shows that a MET needs to be done to find stable, and high-yielding genotypes that are more adaptable and can be used in specific agro-climatic conditions.

Previously, Finlay and Wilkinson (1963) used a number of stability metrics, such as linear regression analysis, as a stability indicator. In GEI, Eberhart and Russell (1966) underlined the significance of incorporating both linear and nonlinear variables when determining the stability of a genotype. Based on this approach, the term “stable genotype” refers to a genotype that behaves uniformly under all studied conditions/environments. Consequently, the stable genotype has a high mean performance (*bi* = 1.0) and the lowest deviations from regression (*S* ^*2*^ *di* = 0). The regression value explains the adaptability of the evaluated genotypes across the assessed environments. The desirable stability required for a genotype is considered as a regression value approaching 1, and a higher mean performance is superior. A genotype having a lower mean performance, a regression value of less than one, and non-significant *S* ^*2*^ *di* does not adapt effectively to favorable environments, and therefore might be marked as a genotype with adaptability to low-yielding environments (Shrestha et al., 2021). On the other hand, genotypes having a higher mean performance, a regression value greater than one, and a non-significant *S* ^*2*^ *di* are considered as low-stable genotype. These groups of genotypes effectively perform across high-yielding conditions but not so well in low-yielding environments. Consequently, they are able to effectively adapt across different conditions (Shrestha et al., 2021). In the case of yield, the genotypes BWL6964, BWL7493, BWL7497, BWL7504, BWL7506, and BWL7511 possess regression values greater than 1, which indicates that they are suited to high-yielding environments, while the genotypes BWL6228, BWL7495, BWL7509, PBW761, PBW725, and HD3086 possess regression values less than 1, which implies that they are suited to low-yielding environments (Table 4). Similar results were also obtained by (Tanin and Gupta, 2018) in Indian mustard and by Shrestha et al. (2021) in maize. For GPC, the genotypes BWL 7493, BWL7495, BWL7504, BWL7508, BWL7509, and BWL7511 had regression values greater than 1, which implied that they adapted to favorable environments, while the genotypes BWL6228, BWL6964, BWL7497, BWL7508, PBW761, PBW725, and HD3086 had regression values less than 1, which confirmed that they are more desirable for unfavorable environments (Table 4).

The article "Ascertaining yield and grain protein content stability in wheat genotypes having the Gpc-B1 gene using univariate, multivariate, and correlation analysis" was published in 2022. Journal: Front Genet.

In this case, the observed variation related to genotype and GEI facilitated the selection process of the ideal genotypes for desired characters, and in such cases, reducing the possible influence of environmental component effects is important (Singh et al., 2019). In this case, the AMMI2 model was considered the most effective analysis pattern to explain the genotypic stability of yield, genomic based variance available among the genotypes, and further provide interesting knowledge regarding the GEI (Oliveira et al., 2014). In addition, if the environments possess smaller IPCA1 and IPCA2 values (near to the origin of biplot), they provide a larger contribution to genotypic stability but contribute a smaller proportion to the GEI (Hilmarsson and Rio, 2021). As a result, ENV2 and ENV4 were the major players in the genotypic stability of grain yield and GPC, respectively. In the AMMI2 biplot, genotypes with the longest distance from the centre of the biplot located near to an evaluated environment are recorded as high-yielding genotypes with great adaptability in such a tested environment (Enyew et al., 2021). In the case of grain yield, the genotypes BWL7495 and BWL7504 were located close to ENV2 in the present study, implying their strong yield potential and greater adaptability specific to this environment as compared to other environments. Similarly, the genotypes BWL6964, BWL7493, and BWL7497 had better performance in ENV6. For GPC, the genotypes BWL7506, and PBW725 were placed close to ENV8, indicating their high GPC potential and better adaptability specific to this environment over other environments. Also, the genotype BWL7493 was observed to have greater GPC performance in ENV3. Whenever different genotypes respond differently to different environments, it strongly suggests the presence of GEI and the existence of variation among environmental components such as soil fertility, precipitation, and temperature. As a result, the selection of wheat genotypes specific to each environment across various agro-climatic conditions is suggested. Environment-specific genotypes with high-yielding and high-GPC potential have already been reported in wheat (Groos et al., 2003; Singh et al., 2019) and other cereal crops (Bantayehu et al., 2011; Solonechnyi et al., 2018).

The article "Ascertaining yield and grain protein content stability in wheat genotypes having the Gpc-B1 gene using univariate, multivariate, and correlation analysis" was published in 2022. Journal: Front Genet.

The “which-won-where” model of GGE biplot was applied to select the top-performing genotypes by explaining the GEI, mega-environment clustering, and environment or genotype specific adaptation (Bishwas et al., 2021; Khan et al., 2021). The genotypes with the longest distance from the origin of biplot are considered the best across all or some of the evaluated environments, and were classified as environment-specific genotypes, because they showed more variation in regards to change in environmental components (Singh et al., 2020). The “which-won-where” model of biplot grouped all the evaluated environments into three and two mega-environments involving different genotypes with high-potential for grain yield and GPC, respectively. In terms of yield, mega-environments 1 contained ENV1, and ENV5 where BWL7506 was considered the best high-yielding genotype, mega-environments 2 contained ENV2, and ENV6 where BWL7493 was recorded as the top yielding genotype, mega-environments 3 contained ENV3, and ENV8, where BWL6228 was observed as the most high-yielding genotype, and mega-environments 4 contained ENV4, and ENV7 where PBW725 was considered the high-performing genotype. On the other hand, for GPC, mega-environment 1 contained only ENV1 where BWL 7509 was observed as the high-GPC genotype, while mega-environment 2 involved ENV2, ENV3, ENV4, ENV5, ENV6, and ENV7 where BWL7511 were recorded as the top-performers, and mega-environment 3 involved only ENV8 where BWL7506 and BWL7508 were observed as top-GPC genotypes. The examined environments were grouped into mega-environments and further identification of mega-environment specific genotypes is the sustainable method to use GEI according to the interests of breeders (Yan and Tinker, 2005). Investigation of mega-environments has been previously reported in different cereals, including wheat (Gerrish et al., 2019), rice (Krishnamurthy et al., 2017), maize (Pererira et al., 2021), and barley (Hernandez-Segundo et al., 2009).

The article "Ascertaining yield and grain protein content stability in wheat genotypes having the Gpc-B1 gene using univariate, multivariate, and correlation analysis" was published in 2022. Journal: Front Genet.

The ranking model of GGE biplot is capable of identifying the high-ranking genotypes with great stability based on AEC decisions (Singh et al., 2020). The AEC based ranking model of biplot recorded the genotypes BWL7497, BWL7506, BWL7508, BWL7511, and PBW725 as the high-ranking for yield, and the genotypes BWL6964, BWL7504, and BWL7508, BWL7509, and BWL7511 as the high-ranking for GPC. However, in the case of yield, the BWL6228, BWL7497, BWL7509, and BWL7511 were recorded as poorly stable genotypes because of the effect of GEI components. Also, for GPC, BWL6228, BWL6964, BWL7497, and BWL7508 were observed as the genotypes with lower stability, which is associated with a GEI effect. Previously published studies on wheat also reported that top-performing genotypes are not always the stable ones (Bassi and Sanchez-Garcia, 2017; Popevic et al., 2020). One of the most useful features of the GGE biplot is the graphical representation of genotypes with the best mean performance and stability. Based on the mean vs. stability model of GGE biplot, the genotypes with the highest AEC prediction (top mean) combined with the shortest stability vector (greatest stability) are considered the best genotypes (Farshadfar et al., 2012; Khan et al., 2021). Accordingly, BWL7508, and BWL7511 were selected as high-performers and highly stable genotypes for yield and GPC. Based on all this, it is concluded that the GGE biplot is the best analysis method as compared with AMMI model for the identification and selection of top genotypes with the most efficient stabilities and the highest performing capabilities. This method has already been used in many studies to identify the top-performing and well-stable genotypes in wheat (Bishwas et al., 2021) and some other cereals, including rice (Mostafavi et al., 2011), maize (Ruswandi et al., 2021) and barley (Ghazvini et al., 2021).

GGE biplot analysis identified the genotypes BWL7497, BWL7506, BWL7508, BWL7511, and PBW725 as the high-yielding and, similarly, BWL6964, BWL7504, BWL7509, and BWL7508, BWL7511 as the top performing genotypes for GPC across all environments. Among all the genotypes, BWL7508, and BWL7511 were selected as ideal genotypes for their great stability, top mean yield, and GPC across all the environments. It is true that these two traits are negatively correlated, but if we deal with a large number of segregants during development of the material, a few lines can be identified combining both GPC and yield. Balancing yield and quality together in a wheat cultivar is a tedious task and can be achieved through some inter-trait trade-offs. The reduction in yield is primarily mediated through a reduction in 1000-grain weight in the *Gpc-B1* positive lines. But in such cases, the number of effective tillers and grins per spike is adjusted to compensate for the yield. A similar result is observed in some previously conducted studies in the wheat germaplasm with Indian origin (Vishwakarma et al., 2014, 2016; Gupta et al., 2022). The present study remarkably identified that the acceptable level of stability and top-performing potential in one genotype for a character are not the same in other characters. This could be due to the role of different genes in the regulation of the different characters or may be because of variation in expression patterns of genes in different genotypes as a direct effect of different environmental factors, such as different abiotic stresses. Several earlier studies have reported similar results in wheat (Du et al., 2020), soybean (Chaves et al., 2017) and rice (Balakrshnan et al., 2016).

The article "Ascertaining yield and grain protein content stability in wheat genotypes having the Gpc-B1 gene using univariate, multivariate, and correlation analysis" was published in 2022. Journal: Front Genet.

In this study, it was found that different univariate, AMMI, and GGE biplot analyses showed somewhat consistent results in terms of the stability potential of the genotypes. The high ranking genotypes were somewhat different, but we selected the genotypes based on their stable performance for both the yield and GPC, and similar results were obtained across all the univariate and multivariate analyses. The AMMI and GGE biplot showed different results in terms of the discriminating potential of environments. As a result, the environments in the AMMI model were closer to the origin than in the GGE biplot. Keeping the discriminating potential of the AMMI model in view, the GGE biplot model is also successfully employed to examine the multi-location data for stability analysis of wheat and rice genotypes (Khan et al., 2021). In the present study, the GGE biplot model observed the genotype and GEI more efficiently as compared to the AMMI model. The same result was recently reported by Khan et al. (2021). Furthermore, in this study, the biplot graph was extremely successful in mega environment classification, identification of representative and discriminative environments, and genotype ranking. A similar result was observed by Oladosu et al. (2017), where the stability performance of rice genotypes was analyzed. The GGE biplot is considered an extremely valuable statistical technique to deeply understand the GEI in a multi-environmental test. However, the decisions for genotypic stability were similar in both the univariate and multivariate analyses. These results are consistent with the results reported in some previously published studies (e.g., Singh et al., 2019; Bishwas et al., 2021). This type of dissimilarity is not avoidable due to different statistical analysis models that were employed in the present study.

The article "Ascertaining yield and grain protein content stability in wheat genotypes having the Gpc-B1 gene using univariate, multivariate, and correlation analysis" was published in 2022. Journal: Front Genet.

## Conclusion

In the present study, a multi-environmental investigation was conducted to evaluate 13 wheat genotypes across different environments to select ideal genotypes. We provided detailed information on the effect of GEI, the stability and adaptability of genotypes to specific environments, and the ability of environments to distinguish between DTF, DTM, PH, SPS, GPS, yield, TGW, and GPC in Punjab State, India. Of these traits, we focused on grain yield and GPC because of their importance to food and nutritional security in the world. These two traits were significantly influenced by environmental, genotype, and GEI effects. Based on the results of this study, it is clearly observed that the wheat near-isogenic lines are the best breeding materials that carry potential variation to improve yield and GPC in wheat. The GGE biplot and AMMI were reported to be the best models to show the effects of GEI in a graph and select the best genotypes with the most adaptability and the best performance. Among the genotypes, BWL7508, and BWL7511 were observed to be highly stable and well performed in terms of yield and GPC across all the environments. In the case of yield, ENV1 and ENV3 were identified as the most representative and discriminating environments for yield, respectively. On the other hand, for GPC, ENV3 and ENV7 were observed to be the most discriminating and representative environments, respectively. Thus, these environments could be further used for the identification of the best genotypes and the selection of high-performing genotypes with environment specific adaptability.

## Data Availability

The original contributions presented in the study are included in the article/Supplementary Material, further inquiries can be directed to the corresponding authors.
